RETRACTED

# The Application of Molecular Techniques for Assessment of SOX2 and miR126 Expression as Prognostic Markers in Esophageal Carcinoma

**DOI:** 10.1155/2022/1514412

**Published:** 2022-02-23

**Authors:** Amal F. Gharib, Wael H. Elsawy, Amani A. Alrehaili, Hanan S. Amin, Hayaa M. Alhuthali, Maha M. Bakhuraysah, Ahmad El Askary

**Affiliations:** ^1^Department of Clinical Laboratory Sciences, College of Applied Medical Sciences, Taif University, P.O.Box 11099, Taif 21944, Saudi Arabia; ^2^Department of Clinical Oncology, Faculty of Medicine, Zagazig University, Egypt; ^3^Department of Clinical Chemistry, Theodor Bilharz Research Institute, Cairo, Egypt

## Abstract

**Objective:**

To study the problem in esophageal cancer, the function of SOX2 and miR-126 has not been completely explored. The objective of this study was to find out how SOX2 and miR-126 act in esophageal cancer and their relation to the clinical and prognostic features.

**Methods:**

The expression of SOX2 and miR-126 was properly assessed in the carcinoma of the esophagus, and the nearby healthy tissues surgically excised from 35 included patients.

**Results:**

SOX2 was elevated in esophageal cancer relative to normal tissues contrary to the miR-126 levels. This inverse relationship was linked to adverse clinical features.

**Background:**

SOX2 has been involved as an oncogene in various types of malignant tumors; microRNA-126 (miR-126) is extensively expressed in vascular endothelial cells, which control angiogenesis. Furthermore, many published reports reasonably concluded that based on the prime characteristic of malignant cells, miR-126 may act appropriately as a promotor or a suppressor for the malignant growth.

**Conclusion:**

In esophageal cancer, SOX2 works as an oncogene, whereas miR-126 acts as a tumor suppressor gene. SOX2 overexpression and miR-126 downregulation were shown to be linked to a poor prognosis.

## 1. Introduction

Carcinoma of the esophagus (CE) is generally rated as the eighth most significant type of cancer and the sixth most common cause of cancer-related deaths [1]. A significant increase in the observed incidence of CE has invariably led to a profound influence on the healthcare system [2].The CE is frequently associated with a poor 5-year survival rate varying from 4% to 40% depending on disease progression, with an overall 5-year survival rate of 18% [3].

MicroRNAs (miRNAs) are small non-coding areas consisted of 20–22 nucleotides in the RNAs; it optimally performs a significant role in mammals by adequately regulating an essential verity of molecular processes [4, 5]. Disturbed regulation of one or a limited number of miRNAs has been appropriately recognized to naturally produce a profound impact on the proper mode of expression of hundreds of mRNAs that pushes resolutely the cells to transform [6, 7]. Several published reports scientifically prove that over 50% of the miRNAs genes are in cancer-associated genomic locations or unstable sites [8, 9]. Genomic expression analysis from an extensive range of malignant tissues/cells showed that the active presence of aberrant miRNA undoubtedly continues to remain a fundamental principle rather than an event [10, 11].

RETRACTED

SOX2 represents an active component of the SRY-related HMG-box (SOX) transcription factor group, which has a wide variety of well-known and complex functions in stem cell proliferation and preservation, embryonic differentiation, and cancer [12, 13].

SOX2 has been naturally involved as an oncogene in various types of malignant tumors like central nervous system (CNS) [14], colorectal [15, 16], melanoma [17, 18], and hepatocellular carcinoma (HCC) [19, 20]. Properly considering its oncogenic activity in many specific types of malignant tumors, however, SOX2 inhibition has been uniquely identified as a key feature of the gastric carcinomas [21, 22].

Increasing evidence indicates precisely that SOX2 represents the principal regulator of stem cell-like cancer cell subgroup, often known to as cancer stem cells (CSCs), which have been promptly reported to be responsible for the neoplastic and invasive abilities for the most types of tumors [23].

Angiogenesis is critical for normal human development, cancer invasive growth, and the pathophysiology of malignant tumors [24, 25]. Angiogenesis is often driven by various signaling pathways and growth factors, including transforming growth factor-beta (TGF-*β*), fibroblast growth factor (FGF), and vascular endothelial growth factor (VEGF), according to several published research [26].

The AKT pathway is one of the most important routes in the malignant process. Cancer develops and spreads as a result of its activation. Overexpression of SOX2 in malignant tumors is dependent on AKT, which phosphorylates it, preventing it from degrading [27].

MicroRNA-126 (miR-126) is accurately located in intron 7 of the epidermal growth factor-like domain 7 (EGFL7) [28] and is extensively expressed in vascular endothelial cells which control angiogenesis by binding to multiple transcripts [29] Furthermore, the published reports of multiple studies have sufficiently shown that the miR-126 is either a tumor suppressor or an oncogene based on the specific type of malignant tumor. Increased levels of miR-126 have been noted in leukemia [30], and diminished miR-126 expression in colorectal adenocarcinoma [31], oral squamous cell carcinoma (OSCC) [32], and lung cancer cell lines [33].

RETRACTED

In esophageal cancer, the function of SOX2 and miR-126 has not been well-investigated. The current study aims to explore at the role of SOX2 and miR-126 in esophageal cancer and their possible association with the clinical and pathological features.

## 2. Patients and Methods

This study was conducted at Zagazig University Hospital, Egypt, between May 2016 and June 2019. It included 35 patients with esophageal cancers who underwent surgery. Informed consent was obtained from all patients in addition to the approval of the ethical committee of Zagazig University. Tissue specimens from the tumor (CE) and nearby healthy tissues (NT) were obtained during surgery from all patients and stored at −80°C in liquid nitrogen until analysis. Patients were clinically staged according to the eighth edition of the American Joint Committee of Cancer (AJCC) [34].

### 2.1. SOX2 and miR-126 Expression by Quantitative Real-Time RT–PCR

#### 2.1.1. RNA Extraction

The total RNA was carefully extracted from the tissue specimens by the Mini Kit miRNeasy purchased from (Qiagen, Hilden, Germany) based on the company instructions. The purified RNA is properly preserved at −80°C until their use.

#### 2.1.2. Complementary DNA (cDNA) Synthesis

Utilizing iNtRON Biotechnology directed by company manuals, extracted RNA was reverse transcripted to synthesize the cDNA.

#### 2.1.3. RT-PCR

The quantitative real-time polymerase chain reaction (qRT-PCR) was performed by SYBR Green PCR Master Mix, Perfect Real-Time purchased from TaKaRa Biotechnology, Japan, based on their instructions.

A total volume of 20 *μ*l amplification solution containing: SYBR Green master mix, 10 *μ*l; 5 *μ*lcDNA; and 100 pmol/*u*l primers was used to run the qRT-PCR by Stratagene, Mx3005P-qPCR. For internal control, glyceraldehyde-3-phosphate dehydrogenase (GAPDH) has been used. The primers used were as follows: (a) GAPDH sense: forward primer, 5′-ACA TGT TCC AAT ATG ATT CC-3′ and reverse primer, 5′-TGG ACT CCA CGA CGT ACT CAG-3′; (b) SOX2: forward primer, 5′-GGGAAATGGGAGGGGTGCAAAAGAGG-3′ and reverse primer, 5′-TTGCGTGAGTGTGGATGGGGATTGGTG-3′; and (c) miR-126: forward primer, 5′-GGA ATG TAA GGA AGT GTG-3′ and reverse primer, 5′-GAG CAG GCT GGA GAA-3′.

The PCR was performed in triplicate, the expression of miR-126 and SOX2 mRNA were normalized to GADPH using the 2^−*ΔΔ*Ct^ calculation [35].

### 2.2. Statistical Analysis

Statistical analysis was performed using the SPSS software version 12.0 for Windows. Student's *t*-test and analysis of variance (ANOVA) test were used to determine if there is a significant difference between the means of studied groups. Pearson's correlation analysis was determined to evaluate the correlation between SOX2 and miR-126 in esophageal cancer tissues.

RETRACTED

## 3. Results

### 3.1. Expression of SOX2 and miR-126 in the Carcinoma of the Esophagus (CE) and the Nearby Healthy Tissues (NT)

The quantitative real time PCR was used to evaluate the mRNA levels of SOX2 and miR-126 in CE and NT obtained from thirty-five patients. In esophageal carcinoma, SOX2 was significantly elevated relative to normal tissues. The mean ± SD was 4.39 ± 0.54 in cancer vs 0.50 ± 0.27 in noncancerous (Figure 1). The difference was statistically significant (*t* = 37.94, *P* < 0.0001). miR-126 was downregulated in the esophageal carcinoma with a mean ± SD of 0.96 ± 0.59 vs 4.22 ± 1.70 in the corresponding normal tissues with a statistically significant difference (*t* = 10.76, *P* < 0.0001). We carefully tested for the practical ability of SOX2 and miR-126 to distinguish CE from NT by plotting the receiver operating curve (ROC). It showed high specificity of both SOX2 and miR-126 with an area under the curve (AUC = 1.00, 95% CI: 1.000 to 1.000, *P* < 0.0001) and (AUC = 0.96, 95% CI: 0.92 to 1.00, *P* < 0.0001), respectively (Figure 2).

SOX2 and miR-126 were assessed in 35 tumor samples and the nearby normal tissues using qRT-PCR. The SOX2 levels were significantly elevated in normal tissues (*t* = 37.94, *P* < 0.0001). miR-126 levels were increased in normal esophageal tissues versus cancerous tissues (*t* = 10.76, *P* < 0.0001).

### 3.2. Correlation between SOX2 and miR-126 in Esophageal Cancer Tissues

Pearson's correlation analysis of the relation between SOX2 and miR-126 in esophageal cancer tissues revealed that increased levels of SOX2 expression were significantly associated with the downregulation of miR-126 (*r* = 0.957, 95% CI: 0.916 to 0.978, *P* < 0.0001) (Figure 3).

When we explored the association between the expression levels SOX2 and miR126 in esophageal cancer tissues, we observed an inverse relationship linking them (*r* = 0.957, 95% CI: 0.916 to 0.978, *P* < 0.0001).

### 3.3. SOX2 And miR-126 Expression and Clinical and Pathological Features in Esophageal Cancer

SOX2 expression measures analysis revealed there was no significant correlation between SOX2 and patient's gender meanwhile, its elevation is significantly related to the cervical or thoracic location, the histopathological type, serum albumin level, the grade of differentiation of tumor, the tumor size, the lymph node involvement, and the clinical stage (Table 1).

miR-126 expression levels were also unrelated to the gender but were significantly related to the location within the esophagus, the histopathological type and grade, the serum albumin level, the tumor size, the lymph node infiltration, and the clinical stage (Table 1).

RETRACTED

## 4. Discussion

Esophageal cancer is still a major health problem all over the world, especially in Asian countries. There is an increasing need to begin precisely to properly look for more effective and useful diagnostic and prognostic molecular markers for this aggressive tumor. miRNAs are short non-coding RNAs that regulate genes at the post-transcription level [4, 6]. Increasing evidence confirms that miRNAs are abnormally expressed in many types of malignant tumors [36].

Tumor-initiating cells or stem-like cancer cells are a group of malignant cells in the tumor tissues that have the ability of self-renewal and diversely differentiate to resistant colonies. They are also involved in promoting metastases and resistance to treatment, thus enhancing cancer growth and recurrence [9, 17]. SOX2 gene is considered one of the key regulators of stem-like cancer cells [37]. miR-126 is involved in the biology of cancer, but its function has not been well-evaluated [38]. The role of SOX2 and miR-126 in esophageal cancer was fully uninvestigated. In the current study, we tried studying their role in esophageal cancer and their relation to clinical and pathological features.

The current study contribution offers proof that the miR-126 was downregulated and SOX2 was elevated in esophageal cancer compared to the normal esophageal tissues. High levels of SOX2 are crucial to providing stem cells like to a variety of malignant tumors [39]. SOX2 was significantly elevated in HCC, colorectal carcinoma, melanoma, and carcinoma of the stomach.

Otsubo et al. published earlier that SOX2 expression was frequently downregulated in human gastric carcinoma, but the underlying mechanism of this downregulation was unreported [14]. Later they reported that miR-126 inhibits the SOX2 mRNA in the cell lines of gastric carcinoma [16]. Our findings support the reports of Otsubo et al. [14]; we found an inverse relationship between elevated levels of SOX2 and downregulation of miR-126. miR-126 is linked to the vascular endothelium and is documented to facilitate angiogenesis [18]. Besides, it was documented to prevent apoptosis in leukemic cells and targeting polo-like kinase 2, which acts as a tumor suppressor promoting colony formation of the progenitor cells in the bone marrow of mice [25]. On the other side, miR-126 was reported previously as a suppressor of tumor growth in colorectal cancer [26]. Whether miR-126 functions as a suppressor or as an oncogenic miRNA, in the present study, we noticed that miR-126 functions as an inhibitor for malignant growth, it was downregulated in malignant relative to normal tissues, and its downregulation was associated with increased SOX2 in tumor tissues, but our results need to be emphasized. Such functional variations in tumorigenesis could be considered a lineage-dependence [33, 34].

RETRACTED

Yang et al. reported that miR-126 inhibits the growth and progression of osteosarcoma cells by targeting SOX2 [35]. More research is required to explore the molecular role of miR-126 in esophageal cancer and other malignancies.

We focused our current research on the possible importance of SOX2 and miR-126 as molecular markers for prognosis in esophageal carcinoma, the upregulation of SOX2, and the downregulation of miR-126 was linked to adverse clinical and prognostic features. The upregulation of SOX2 and downregulation of miR-126 in esophageal carcinoma was related to the location, histopathologic type, grade, size, and stage of tumor in addition to the serum albumin level and the presence of lymph node infiltration. These results agree with the previously published reports in several malignant tumors.

In conclusion, the current study showed that miR-126 behaves as a tumor suppressor in carcinoma of the esophagus. Our results also revealed that miR-126 and SOX2 could be used as biological markers to predict the prognosis in esophageal carcinoma.

## Figures and Tables

**Figure 1:** SOX2 mRNA expression and miR-126 expression in normal and esophageal carcinoma tissues.

**Figure 2:** A receiver operating characteristic curve (ROC) of SOX2 (a) and miR-126 (b) in esophageal cancer tissues (EC). ROC revealed a high specificity of SOX2 and miR-126 for ECT (AUC = 1.00, 95% CI: 1.000 to 1.000, *P* < 0.0001) and (AUC = 0.96, 95% CI: 0.92 to 1.00, *P* < 0.0001), respectively.

**Figure 3:** Pearson's correlation between the expression of SOX2 and miR-126 in esophageal cancer tissues. A significant association between the increased SOX2 levels and the downregulation of miR-126 (*r* = 0.957, 95% CI: 0.916 to 0.978, *P* < 0.0001).

**Table 1:** SOX2 and miR-126 expression and clinical and pathological data.

		miR-126		P	SOX2		P
	*n*	Mean	SD		Mean	SD	
Sex							
Male	30	0.95	0.57	0.81^∗^	4.39	0.55	0.91^∗^
Female	5	1.02	0.78		4.36	0.57	
Location							
Cervical	5	1.71	0.09	<0.00	5.21	0.22	<0.0001^∗∗^
Thoracic	17	1.22	0.37	01^∗∗^	4.59	0.20	
Abdominal	13	0.33	0.23		3.80	0.20	
Pathology							
Adeno^a^	20	1.17	0.58	0.010	4.60	0.57	0.0045^∗^
SCC^b^	15	0.67	0.48	1^∗^	4.10	0.34	
Albumin, g/dl							
≤3.7	15	1.56	0.15	<0.00	4.88	0.28	<0.0001^∗^
>3.7	20	0.51	0.33	01^∗^	4.02	0.36	
Grade							
I	12	1.62	0.11	<0.00	4.94	0.28	<0.0001^∗∗^
II	10	0.98	0.30	01^∗∗^	4.48	0.17	
III	8	0.47	0.17		3.93	0.03	
IV	5	0.10	0.07		3.59	0.16	
T							
T1	12	1.62	0.11	<0.00	4.94	0.28	<0.0001^∗∗^
T2	7	1.11	0.26	01^∗∗^	4.58	0.07	
T3	10	0.56	0.15		4.04	0.17	
T4	6	0.13	0.08		3.63	0.19	
N							
N0	13	1.6	0.12	<0.00	4.9	0.3	<0.0001^∗∗^
N1	16	0.75	0.31	01^∗∗^	4.2	0.3	
N2	6	0.13	0.08		3.6	0.2	
Stage							
I	14	1.58	0.13	<0.00	4.90	0.28	<0.0001^∗∗^
II	15	0.57	0.22	01^∗∗^	4.11	0.26	
III	6	0.47	0.60		3.89	0.57	

^a^Adenocarcinoma, ^b^squamous cell carcinoma, and ^∗^Student's *t*-test. ^∗∗^Analysis of variance (ANOVA).

RETRACTED

## Data Availability

The data of the present study are available on request.
